RETRACTED

# IoT-Oriented Wireless Sensor Network and Sports Dance Movement Perception

**DOI:** 10.1155/2022/6477170

**Published:** 2022-09-30

**Authors:** Lin Zhu

**Affiliations:** College of Arts, Wuhan Sports University, Hubei, Wuhan 430079, China

## Abstract

The Internet of Things needs to connect different types of sensors in accordance with the agreement, and different agreements can be used for information and information exchange systems, which can facilitate the identification and control of intelligent systems. In many scenarios, location service application data are very important for obtaining accurate location information about nodes. In this paper, a wrist motion sensing sensor based on the PVDF piezoelectric film is developed. To realize the monitoring of wrist motion signals, this paper designs and manufactures a series of PVDF noninvasive sensors for motion perception. The characteristics of sports dance movements are reflected in the coordination between men and women, and the dance posture and movements must be synchronized with the music according to the level of music rhythm structure. The transfer of center of gravity is the main driving force of sports, and the gait of athletes is related to the transfer of center of gravity. Posture stability is the basic element of sports dance training. Only on this basis can it be possible to develop specific motion function trajectories and technical action forms.

## 1. Introduction

The Internet of Things has certain development prospects in some broad fields, and each positioning information needs to be accurately found. In many scenarios, location service application data are very important for obtaining accurate location information about the site [1]. Therefore, the research on precise positioning of the Internet of Things has a great social and commercial significance; for individuals, it can also effectively improve the quality of life [2]. Based on the in-depth study on the research results of the positioning algorithm of the Internet of Things, the improvement of the positioning algorithm can further improve the positioning accuracy [3]. The Internet of Things expands based on the Internet [4], connecting people, people and things, and things with things [5]. With the continuous development of the Internet of Things, sensors have been applied more and more [6]. In some applications, location information is very important, and the data used can only be effective if it contains appropriate location information. Generally speaking, the development of a high-precision, low-complexity wireless sensor network positioning algorithm has always been an urgent need in the field of wireless research [7]. Technical problems are solved. This article takes some equipment as a starting point and then starts with the design of each unit to realize the detection of each motion signal. Investigate and study some key issues in the PVDF sensor array developed [8]. The ultimate goal of this article is to detect motion signals, use gesture recognition algorithms to realize finger motion perception, design and manufacture a set of PVDF sensor array devices, and provide a new and convenient human-computer interaction device for man-machines [9, 10]. This article does not study the hand movements because according to the sports dance technique, the standard dance arm is a fixed frame type, and different dance movements are issued by the dance arm of the body, passing through the shoulder and foot bones to the terminal fingers and then become the most basic law of movement. The limitation of the quality of sports dance technical movements comes from the results of competitive attributes, evaluation standards, and music. The environmental limitations of sports dance technical movements come from the rules of the competition and the competition venue. As a background venue for performing technical moves, athletes can fully participate so that referees can conduct objective and rational analysis. When the quality of a technical action can be observed, it is difficult to describe its parts individually. All the athletes' technical actions must have an “obvious” effect, and any rational analysis by the referee is based on a certain “phenomenon.”

RETRACTED

## 2. Related Works

According to the literature, sports dance training should not only solve the kinematics and dynamics of personal technical movements at any time but also cooperate with dance partners, music, and dance style and express emotions and show themselves [11]. Under many restrictive conditions, the above elements outside the human body are deeply combined with athletes' body movements and artistic expression to show the quality of technical movements, and the pursuit of perfect technical movement quality is the competition content and winning goal [12]. The literature points out that an important technical feature of sports dance and the important feature of human independence is to rely on movement. The beginning of sports dance is reflected in the cooperation between men and women, which is mainly divided into two aspects: gait and center of gravity displacement [13]. Literature review shows that the direct research on “technical movement quality of sports dance” is extremely limited, and there is no corresponding theoretical framework to follow. The literature shows that the famous manipulator and experts in the United States have created bionic technology and can control technology in the development and design of exoskeleton robots [14]. With the rapid development of data, exoskeleton robots have developed rapidly in various countries. However, due to the gap between technology and economic level, the development of robot exoskeleton technology also varies from country to country [15]. The literature briefly introduces the current development and research results of global exoskeleton robot technology. Compared with much foreign exoskeleton technology research, the research and development of foreign skeleton robots lags behind. With the support of technology development and policy environment, action recognition technology has been greatly improved [16].

RETRACTED

## 3. Internet of Things Algorithms and Wireless Sensor Network Application

### 3.1. Internet of Things Algorithm

Based on the positioning algorithm to measure the nodes in some positions, the initial position starts to use the weighted least square method to calculate the estimated value of the problem. Different algorithms have different functions in the positioning of the nodes in the plane.

Different nodal coordinate formulas can be obtained by three-side measurement, such as formulas (1)–(3):

(1) $$\begin{array}{c} {\left(x_{it}-u_{t_{1}}\right)}^{2}+{\left(y_{it}-v_{t_{1}}\right)}^{2}=d_{i,t_{1}}^{2}, \end{array}$$

(2) $$\begin{array}{c} {\left(x_{it}-u_{t_{2}}\right)}^{2}+{\left(y_{it}-v_{t_{2}}\right)}^{2}=d_{i,t_{2}}^{2}, \end{array}$$

(3) $$\begin{array}{c} {\left(x_{it}-u_{t_{3}}\right)}^{2}+{\left(y_{it}-v_{t_{3}}\right)}^{2}=d_{i,t_{3}}^{2}. \end{array}$$

In formulas (4) and (5), (b) minus (a) and (c) minus (b) is the equation set as follows:

(4) $$\begin{array}{c} 2\left(u_{t_{1}}-u_{t_{2}}\right)x_{it}+2\left(v_{t_{1}}-v_{t_{2}}\right)y_{it}=d_{i,t_{2}}^{2}-d_{i,t_{1}}^{2}+u_{t_{1}}^{2}+v_{t_{1}}^{2}-u_{t_{2}}^{2}-v_{t_{2}}^{2}, \end{array}$$

(5) $$\begin{array}{c} 2\left(u_{2}-u_{t_{3}}\right)x_{it}+2\left(v_{t_{2}}-v_{t_{3}}\right)y_{it}=d_{i,t_{3}}^{2}-d_{i,t_{2}}^{2}+u_{t_{2}}^{2}+v_{t_{2}}^{2}-u_{t_{3}}^{2}-v_{t_{3}}^{2}. \end{array}$$

The *T*-th guess of the *I*-th unknown node is

(6) $$\begin{array}{c} \left[\begin{array}{c} x_{it}\\ y_{it} \end{array}\right]={\left[\begin{array}{cc} 2\left(u_{t_{1}}-u_{t_{2}}\right) & 2\left(v_{t_{1}}-v_{t_{2}}\right)\\ 2\left(u_{t_{2}}-u_{t_{3}}\right) & 2\left(v_{t_{1}}-v_{t_{2}}\right) \end{array}\right]}^{-1}\times \left[\begin{array}{c} d_{i,t_{2}}^{2}-d_{i,t_{1}}^{2}+u_{t_{1}}^{2}+v_{t_{1}}^{2}-u_{t_{2}}^{2}-v_{t_{2}}^{2}\\ d_{i,t_{3}}^{2}-d_{i,t_{2}}^{2}+u_{t_{2}}^{2}+v_{t_{2}}^{2}-u_{t_{3}}^{2}-v_{t_{3}}^{2}\; \end{array}\right]. \end{array}$$

Taking each average value as the initial value of *i* position nodes and then we get the estimated value as

(7) $$\begin{array}{c} \left[\begin{array}{c} {\hat{x}}_{i}\\ {\hat{y}}_{i} \end{array}\right]={\left[\begin{array}{cc} \overset{N}{\underset{t=1}{\sum }}x_{it} & \overset{N}{\underset{t=1}{\sum }}y_{it}\\ \bar{N} & \bar{N} \end{array}\right]}^{T}. \end{array}$$

Different positioning models will be expanded to determine the initial value of the position based on the description of the node, the distance between the nodes, and the known information measured by the TOA sorting technology, such as

(8) $$\begin{array}{c} D=Q∆+E. \end{array}$$

Using the weighted least square method to determine the position deviation, we get

(9) $$\begin{array}{c} \left[\begin{array}{c} ∆x_{1}\\ ∆y_{1}\\ \begin{array}{c} \vdots \\ \begin{array}{c} ∆x_{n}\\ ∆y_{n} \end{array} \end{array} \end{array}\right]={\left(Q^{T}T^{-1}Q\right)}^{-1}Q^{T}T^{-1}D. \end{array}$$

According to the process of the algorithm, the time complexity of the algorithm is calculated. On the basis of the Taylor formula, the three-sided complexity of each measurement method is compared, and the value of the number of different nodes is *n*, and each improved three-sided complexity of the edge measurement algorithm is greater than that of other algorithms. The main reason is that the distance of the unknown node increases, which leads to the expansion of the Taylor series, in exchange for higher positioning accuracy. The comparison of time complexity is shown in Table 1.

RETRACTED

Constructing the Fisher information matrix can get formula:

(10) $$\begin{array}{c} F=\left[\begin{array}{cc} F_{xx} & F_{xy}\\ F_{xy}^{T} & F_{yy} \end{array}\right]. \end{array}$$

Equation (11) finds the *F* matrix that satisfies the root mean square error of the positioning result as

(11) $$\begin{array}{c} E\left(\left(\hat{\varphi }-\varphi \right){\left(\hat{\varphi }-\varphi \right)}^{T}\right)\geq CRLB\left(\hat{\varphi }\right)=tr\left(F^{-1}\right). \end{array}$$

When different algorithms are used to verify the validity of knowledge, it is necessary to use simulation technology for simulation calculation, and then determine the positioning algorithm of the trilateration in the Taylor series. The modeling parameter is an area of 100 m × 100 m, 20 nodes are randomly and uniformly distributed, and simulated independently for 1000 times. Formula 12 can be obtained as

(12) $$\begin{array}{c} error=\sqrt{E\left(\overset{n}{\underset{i=1}{\sum }}{\left(\tilde{x_{i}}-x_{i}\right)}^{2}+{\left(\tilde{y_{i}}-y_{i}\right)}^{2}\right)}. \end{array}$$

Based on the different initial values of the positioning algorithm, it is necessary to use the least square method to estimate each different position, and then obtain each environment suitable for the two-dimensional plane.

RETRACTED

The specific steps to solve the positioning algorithm are as follows:

① Establish the distance square matrix, as
  (13) $$\begin{array}{c} D=\left[\begin{array}{cccc} 0 & d_{1.2}^{2} & \cdots & d_{1.\left(n+m\right)}^{2}\\ d_{1.2}^{2} & 0 & \cdots & d_{2.\left(n+m\right)}^{2}\\ \vdots & \vdots & \ddots & \vdots \\ d_{1.\left(n+m\right)}^{2} & d_{2.\left(n+m\right)}^{2} & \cdots & 0 \end{array}\right]. \end{array}$$
② After each different center matrix is determined, multiply, then we get
  (14) $$\begin{array}{c} J=E-{\left(n+m\right)}^{-1}.I. \end{array}$$

The matrix *H* after double centralization has the form

(15) $$\begin{array}{c} H=-\frac{1}{2}JDJ. \end{array}$$

After the determination of different initial positions, the position of the anchor node and the distance between the two are measured using TOA sorting technology. Different Taylor set formulas create different models between multivariate expansions, and then we get

(16) $$\begin{array}{c} D=Q∆+E. \end{array}$$

Equation (17) uses the least square method to solve the position deviation:

(17) $$\begin{array}{c} \left[\begin{array}{c} ∆x_{1}\\ ∆y_{1}\\ \begin{array}{c} \vdots \\ \begin{array}{c} ∆x_{n}\\ ∆y_{n} \end{array} \end{array} \end{array}\right]={\left(Q^{T}Q\right)}^{-1}Q^{T}D. \end{array}$$

Equation (18) is the estimated location of the unknown node:

(18) $$\begin{array}{c} \left[\begin{array}{c} \tilde{x_{1}}\\ \begin{array}{c} \tilde{y_{1}}\\ \vdots \\ \begin{array}{c} \tilde{x_{n}}\\ \tilde{y_{n}} \end{array} \end{array} \end{array}\right]=\left[\begin{array}{c} \hat{x_{1}}+∆x_{1}\\ \begin{array}{c} \hat{y_{1}}+∆y_{1}\\ \vdots \\ \begin{array}{c} \hat{x_{n}}+∆x_{n}\\ \hat{y_{n}}+∆y_{n} \end{array} \end{array} \end{array}\right]. \end{array}$$

The output mode of CRLB needs to be based on a certain algorithm in each positioning algorithm, and then meet the error according to the positioning as

(19) $$\begin{array}{c} E\left(\left(\hat{\varphi }-\varphi \right){\left(\hat{\varphi }-\varphi \right)}^{T}\right)\geq CRLB\left(\hat{\varphi }\right)=tr\left(F^{-1}\right). \end{array}$$

When the measured error is zero, the variance can be determined as an estimate of performance, and the Gaussian distribution of the root mean square error can be determined. Looking for the positioning algorithm, we obtain

(20) $$\begin{array}{c} error=\sqrt{E\left(\overset{n}{\underset{i=1}{\sum }}{\left(\tilde{x_{i}}-x_{i}\right)}^{2}+{\left(\tilde{y_{i}}-y_{i}\right)}^{2}\right).} \end{array}$$

### 3.2. Wireless Sensor Network Application

Because some higher-dimensional two-dimensional spaces are more intuitive, you only need to consider the two-dimensional situation. In the two-dimensional situation, the position information of the wireless sensor node is represented by a column vector of coordinate elements as

(21) $$\begin{array}{c} v_{ij}=\left\{\begin{array}{cc} 1\text{,} & measurable\;situation\text{,}\\ 0\text{,} & other. \end{array}\right. \end{array}$$

The distance between all pairs of nodes is measured as

(22) $$\begin{array}{c} r_{ij}=\left\|p_{i}-p_{j}\right\|+n_{ij},i=1,\ldots ,M,j=1,\ldots ,M,i<j. \end{array}$$

One technique that can be used to reasonably estimate its positioning performance is the AM positioning error of all detected sensor nodes as

(23) $$\begin{array}{c} a.m.s.locazation\;error=\frac{1}{M_{loesen\;}m\in S}\sum E\left\{{\left\|\hat{p_{m}}-p_{m}\right\|}^{2}\right\}. \end{array}$$

According to the CRLB of AMS, formula (24) can be obtained as

(24) $$\begin{array}{c} {CRLB}_{e}=TR\left\{I_{e}^{-1}\right\}. \end{array}$$

The probability density function associated with an independent model of Gaussian measurement error with zero mean and proportional variance is

(25) $$\begin{array}{c} f_{p}\left(r_{ij},i=1,\ldots ,M,j=1,\ldots M,i<j|p_{m},m=1,\ldots ,M\right). \end{array}$$

RETRACTED

## 4. Sports Dance Movement Quality and Movement Perception

### 4.1. Research on the Quality of Sports Dance Movements

The quality of the technical movements of sports dance is not only related to different cognitions of technical knowledge but also related to the performance of body movements. Different sports activities combine different functions in terms of concepts and principles of movement control. In training, one of the movement techniques of each athlete is to include some trajectories, timing, and movement postures related to speed, strength, and rhythm. However, it turns out that time, speed, and rhythm are all part of the content of time, and strength is related to the use of body energy. At the biological level, the understanding of movement is not only from the perspective of movement control theory, but starting from the right phase of human beings, different body movements are connected with the activities of the brain. When each athlete pursues the goal of the competition, he must constantly feel, experience, and create a state of complete or even extreme mobilization and activation of the nervous system. Human gait can be divided into standing period and swing period. The normal gait support in dance movements requires vertical force (floor reaction force) to resist gravity, support body weight, and generate horizontal friction to resist the support surface (to make the body move towards all directions). Need to move in direction. In addition, the posture control strategy needs to be adjusted to make it more flexible, and the speed change and direction also need to be changed. In the change of each support surface, the principle of motion control will complete a certain posture control so that different speed changes can be changed. The basic principle of movement is also based on the training and application of sports dance movement. The athlete's gait model needs new adaptation, especially facing various complex tasks and environmental conditions.

RETRACTED

As a spatial component of the quality of technical movements, the most important function of trajectory and movement methods is to control the body and prepare for the victory of the game. It can reflect the beauty more than art sports and other competitive sports. Therefore, this article examines the relationship between the quality of technical movements and the athletes and space from the perspective of kinematics, and whether the form and trajectory of the movements are related to posture positioning. Technical actions are based on body anatomy and vertical body lines and movement in spherical space. Whether it is basic movements or the movements of standing, walking, running, jumping, turning, and bending, the control of balance is a complex sensation and movement technique. Always keep this in mind during training and take the initiative to adapt to various changes. It is necessary to know that “the space where the body is located will affect the perception of position stability and direction.” Posture stability is the basic element of sports dance sports training. Only on this basis can it be possible to develop specific motor function trajectories and technical movements. Amplitude, acceleration, and speed are a special technical action mode, and they are the external effect components of “mass.”

### 4.2. The Perception of Lower Limb Movement in Sports Dance

The movement of the lower limbs of the human body contains many aspects and types of data although the use of muscle electrical signals can directly reflect the advantages of the brain's muscular awareness of the human body's actions and quickly reflect a person's movement intention. In addition, due to the uncertainty of the environment, the surface EMG signal is also more susceptible to interference. Different surface area signals are used to determine changes in motion status and ensure the accuracy and reliability of body motion. Based on the above considerations, this article assists the inertia and inertia of the lower limbs. Foot pressure information perceives movement behavior and strives to rely on the combination of multiple sports information to make lower limb movement research more accurate and reliable, as shown in Figure 1.

RETRACTED

Taking the lateral thigh muscles as an example, using the above-mentioned method of detecting the end point of the activity segment of the EMG signal can better identify the end point of the activity of the EMG signal, as shown in Figure 2.

After recording the acceleration characteristics, sEMG, and plantar pressure signals separately, some important characteristics can be obtained, but this also leads to an increase in the size of the elements, and the excess elements are also different. Therefore, the preliminary merge function should be checked. This article uses a method to check the relevance and redundancy of the function, as shown in Figure 3.

Table 2 shows the comparison and analysis results of the classification effect data. From the results obtained, the classification accuracy of the algorithm combining the three types of information functions is compared with the method of a single sensor function and compared with the previous method using the gait periodic function as the unit. Compared with the recognition method, the classification accuracy is higher, and at the same time, it has a great advantage in classification efficiency.

## 5. Conclusion

This article aims to further reduce the influence of ranging error on positioning accuracy and improve the positioning accuracy of the algorithm. Based on the Taylor series expansion method, in each of the expansion positioning models, which are mostly Taylor series, each model proposes two brand new positioning algorithms, which combine the multilateral measurement methods, and then uses the MATLAB algorithm to model and test the algorithm. In order to be able to model and analyze the positioning algorithm more intuitively and conveniently, this paper also uses MATLAB to design and implement an IoT node positioning modeling platform. Different environmental monitoring has attracted widespread attention in areas such as intelligent transportation and technological battlefields. Different industrial production and life have gradually expanded to social life. However, as a continuously developing technology industry, it is still in application. As the core technology of WSNS, WSNS positioning technology has always been a research topic for scientific research institutes and enterprises at home and abroad. Different positioning algorithms emerge in endlessly, but no one positioning algorithm is omnipotent and suitable for all situations. Each algorithm has its own advantages and limitations in a given environment. Based on the analysis of the principles and performance of various positioning algorithms, this article assumes the basic requirements of low computing power and high practical feasibility of the product to develop a system that uses a small number of reference nodes. The practice of multiple scenarios requires in-depth research and positioning. Technology and algorithm goals apply part of the positioning information to the real wireless temperature monitoring system. It is the internal and external sum of technical knowledge and performance behavior concepts. It includes many factors, and only when the requirements of these factors are fully met as much as possible will it affect the quality of technical actions.

RETRACTED

## Figures and Tables

**Figure 1:** Low-pass filtering of plantar pressure.

**Figure 2:** Schematic diagram of active segment extraction.

**Figure 3:** Flow chart of the forward search algorithm based on dynamic correlation and redundancy analysis.

**Table 1:** Comparison of time complexity.

Algorithm	Time complexity
Trilateral calculation	O(nm^3^)
Three-sided calculation and traditional Taylor series expansion	O(nm^3^)+O(nm)
Three-sided calculation and Taylor series expansion of multivariate variables	O(nm^3^)+O(n^4^)

**Table 2:** Comparison of three feature classification results.

	Walk (%)	Jump (%)	Raise leg (%)	Stretch (%)
Original period unit	90.12	89.10	92.50	89.98
sEMG	81.32	82.50	89.00	81.20
Acceleration	87.30	87.20	83.92	86.17
Plantar pressure	90.35	91.50	78.65	77.15
Fusion feature	88.93	93.80	91.32	91.56

## Data Availability

The data used to support the findings of this study are available from the corresponding author upon request.
